The article "Analysis of Fast-Track Surgery with Pain Care on Postoperative Pain Improvement and Complication Prevention in Perioperative Spine Surgery Patients" was published in 2022. Journal: Emerg Med Int.

# Analysis of Fast-Track Surgery with Pain Care on Postoperative Pain Improvement and Complication Prevention in Perioperative Spine Surgery Patients

**DOI:** 10.1155/2022/9291583

**Published:** 2022-08-05

**Authors:** Guiyu Xie, Fan Liu, Li Fan, Yi Wen

**Affiliations:** Department of Orthopedics, Foshan Hospital of Traditional Chinese Medicine (Spinal Surgery), Foshan 528000, Guangdong, China

## Abstract

**Objective:**

The study aimed to analyze the effect of fast-track surgery with pain care on the improvement of postoperative pain and the prevention of postoperative complications in perioperative spinal surgery patients.

**Methods:**

A total of 126 patients undergoing spinal surgery from January 2021 to September 2021 were chosen as the study population, and the patients were classified into the regular group, the FTS group, and the combined group by random grouping, with 42 cases in each group. Patients in the regular group used routine perioperative care in spine surgery, patients in the FTS group used the FTS care model, and patients in the combined group combined special pain care on the basis of the FTS group. We compared the numeric rating scale (NRS) and pain severity of patients in the three groups post-op, 30 min, 1 h, 3 h, 6 h, and 24 h after surgery; we compared the time to get out of bed, length of stay, and occurrence of postoperative adverse effects in the three groups, compared the incidence of complications in the three groups, and compared the satisfaction of care in the three groups.

**Results:**

The NRS scores at 12 h, 24 h, 48 h, and 72 h post-op in the combined group and FTS group were lower than those in the regular group, and the NRS scores at 12 h and 24 h post-op in the combined group were lower than those in the FTS group (all *P* < 0.05); the post-op bed activity time, post-op hospitalization time, post-op adverse reaction rate, and post-op complication rate in the combined group and FTS group were shorter or lower than those of the regular group. Nursing satisfaction was higher than that of the regular group, the post-op time to bed activity in the combined group was shorter than that of the FTS group, and nursing satisfaction was higher than that of the FTS group (all *P* < 0.05).

**Conclusion:**

The use of FTS with pain care interventions helps relieve postoperative pain in perioperative patients in spine surgery, reduce the incidence of post-op adverse effects and complications in patients, accelerate their postoperative recovery, and improve nursing satisfaction.

## 1. Introduction

Spine disease is one of the most common diseases in surgery, with the neck and shoulder pain, vertigo, and headache as the main clinical manifestations, and some patients may also suffer from lower limb pain due to involvement, unable to walk upright, or even paralysis in the severe cases, which has adverse effects on the quality of life of patients [1, 2]. In recent years, due to the interaction of a variety of factors, the incidence of spinal diseases increases year by year, and the clinical treatment of spinal diseases has become the main focus of attention [3]. Currently, drugs and surgery are usually used to treat spinal diseases. Drugs can play a certain role in the treatment of mild lesions, but surgery is required for severe spinal diseases [4, 5].

The article "Analysis of Fast-Track Surgery with Pain Care on Postoperative Pain Improvement and Complication Prevention in Perioperative Spine Surgery Patients" was published in 2022. Journal: Emerg Med Int.

However, under the influence of spinal nerve compression, surgical operations, and local inflammatory factor stimulation, patients undergoing spinal surgery often have pain symptoms to different degrees after operation. It is well known that pain refers to an unpleasant sensory and emotional experience of various nociceptive stimuli in the body and abroad, which can cause a series of adverse effects on the patient's body and psyche, reduce the quality of life, and affect the patient's recovery process [6, 7]. Therefore, how to relieve postoperative pain and improve the quality of life is of paramount importance [8]. Postoperative nursing intervention is an important measure to ensure the therapeutic effect [9]. Fast-track surgery (FTS) is one of the widely used nursing modes. It mainly uses the perioperative optimization measures confirmed by evidence-based medicine to help patients reduce stress and prevent postoperative dysfunction [10]. However, clinical practice found that the nursing effect of using FTS alone for surgical patients was limited [11, 12]. Studies have pointed out that FTS care for patients undergoing spinal surgery combined with other optimized care modes may have a positive impact on improving the patients' postoperative recovery. Based on this, we have explored the implementation of FTS combined with pain-specific care for patients undergoing spinal surgery and its effect and impact on the patients' quality of life in the perioperative period and have gained some experience, which is reported in the following sections.

## 2. Data and Methods

### 2.1. General Data

The subjects included in this study were all patients admitted for surgical treatment of the spine from January 2021 to September 2021, with a total of 126 cases. The consent randomized equal division into the regular group, FTS group, and combined group. There is no significant difference in general data such as gender, age, operation time, and body mass index between the three groups (*P* > 0.05), which is comparable.

### 2.2. Inclusion Criteria

Inclusion criteria were as follows: all patients had obvious signs of spinal injury and were diagnosed by examination. All patients met the surgical indications. Patients aged 18 to 65 years; patients with normal cognitive function, understanding the interpretation of the relevant scales by the medical staff, and being able to cooperate with the completion of the assessment of the relevant scales.

The article "Analysis of Fast-Track Surgery with Pain Care on Postoperative Pain Improvement and Complication Prevention in Perioperative Spine Surgery Patients" was published in 2022. Journal: Emerg Med Int.

### 2.3. Exclusion Criteria

Exclusion criteria were as follows: patients with concomitant fractures and obvious painful injuries at other sites; those with the presence of serious cardiovascular, pulmonary, hepatic, renal, respiratory, hematologic, and neurologic diseases, and other diseases affecting postoperative rehabilitation; those with compound spinal injuries; those with coagulation disorders.

### 2.4. Care methods

#### 2.4.1. Regular Group

Patients in the regular care group received only conventional nursing interventions, mainly including nursing staff administered analgesic drugs according to medical prescriptions and analyzed and evaluated the analgesic effect of patients. Patients were given routine health education one day before surgery and were prepared for surgery. The rehabilitation of patients and the prevention of complications were observed after operation.

#### 2.4.2. FTS Group

Patients were cared for on the basis of conventional care combined with the FTS concept. The content of routine care was the same as that of the regular group, and the content of FTS management was as follows: ① formation of the FTS management group: the head nurse of the department was the team leader, and the nursing staff of the department were the team members. The head nurse and the chief surgeon regularly trained the team members on day surgery operation, day surgery nursing cooperation, and FTS-related knowledge and nursing skills. ② Pre-op care: responsible nurses educate patients about disease-related knowledge, surgical procedures, perioperative precautions, postoperative FTS concepts, pain care, etc., before the hospitalization and before surgery. In health education, nursing staff encouraged and affirmed the patients and improved their emotions and treatment compliance through positive psychological suggestion. At the same time, the successful cases of surgical treatment were listed to reduce patients' tension, anxiety, and other negative emotions ③Intra-op care: intra-op warming blankets were given to the patients to keep them warm, and the input fluid and rinse solution should be warmed to 37°C; the amount of intraoperative infusion should be controlled. ④Fast postoperative rehabilitation care: patients needed to receive analgesic care as prescribed by the doctor 3 d after surgery, and the patient's pain level was assessed and analyzed using the numerical assessment method; the attending physician needed to add analgesic medication according to the actual situation of the patient. Patients were allowed to drink a little warm water 4 h after surgery and to eat a little liquid or semiliquid food if they did not have any adverse reaction such as nausea and vomiting within 30 min. In the early postoperative period, patients were encouraged to try to get out of bed for moderate activities, and the amount of exercise could be gradually increased according to their recovery status.

The article "Analysis of Fast-Track Surgery with Pain Care on Postoperative Pain Improvement and Complication Prevention in Perioperative Spine Surgery Patients" was published in 2022. Journal: Emerg Med Int.

#### 2.4.3. Combined Group

The combined group combined pain special nursing on the basis of the FTS group, including the following measures: ①pain education was performed by distributing education manuals, watching videos, and attending a pain salon. Pain education can correct the misconception that patients must bear the pain, so that patients can enhance the sense of pain control, and eliminate the fear, anxiety, and helplessness of pain. It enables patients to understand and master the assessment method of pain severity, report pain timely and accurately, and facilitate timely and effective treatment of pain and discomfort. At the same time, it can help patients correctly understand the pain, alleviate their inner fear and tension, and relieve psychological pressure. Besides, music therapy and suggestion therapy were adopted to distract the patients' attention and help them maintain a relaxed and happy mood and raise pain threshold. The patients were also taught to take deep breaths and meditate to relieve pain. ②Drug analgesic care: the formulation of analgesic treatment plan should be based on the patient's age, health status, expected postoperative pain level, etc., to select the appropriate drug type, dose, route of administration and time so as to achieve the best analgesic effect with the smallest dose. For example, mild pain could be diverted by playing light music, guiding reading, and reading newspapers to reduce their pain level. For moderate pain, alternating hot and cold wet compresses with 50% magnesium sulfate can be applied for 15 min each time, 2∼3 times a day; for patients with severe pain, intramuscular injection of parecoxib 40 mg can be administered twice a day for 3 d, while an intravenous self-administered analgesic pump is applied for 48 h of continuous treatment.

### 2.5. Observation Indexes

#### 2.5.1. Postoperative Rehabilitation-Related Indexes

The postoperative bed activity time, hospitalization time, and occurrence of postoperative adverse reactions were compared between the two groups.

The article "Analysis of Fast-Track Surgery with Pain Care on Postoperative Pain Improvement and Complication Prevention in Perioperative Spine Surgery Patients" was published in 2022. Journal: Emerg Med Int.

#### 2.5.2. Pain Scores and Degrees at Different times

Patients' pain conditions were assessed by the numeric rating scale (NRS), and different degrees of pain were indicated by scores from 0 to 10, where 0 indicated no pain, 1 to 3 indicated mild pain, >3 to 6 indicated moderate pain, and >6 to 10 indicated severe pain. The pain scores and pain severity of the three groups of patients at the time of admission, 24, 48, and 7 2 h after surgery were recorded.

#### 2.5.3. Complications

The occurrence of complications such as postoperative bleeding, postoperative pressure sores, urinary retention, and incisional infections were recorded and compared between the two groups.

#### 2.5.4. Satisfaction with Nursing Care

On the day of discharge, a survey was conducted using our homemade nursing satisfaction survey scale, which consisted of 25 items with individual scores ranging from 1 to 4, and a total score of 100, with higher scores indicating higher patient satisfaction with nursing care. A score of ≥90 was considered satisfactory, a score of 70–89 was considered more satisfactory, and a score of <70 was considered unsatisfactory. Satisfaction = number of cases (satisfied + more satisfied)/total number of cases × 100%.

### 2.6. Statistical Analysis

Statistical software SPSS 18.0 was used to analyze the data, and the mean ± standard deviation (mean ± SD) was used to express the measurement data; the *t*-test was used to compare the age, operation time, BMI, hospital stay, NRS score, and postoperative venting time between the two groups; the *χ*^*2*^ test was used to compare the gender, satisfaction, and complications between the groups, and the pain level was used to compare the groups. Fisher's exact probability test was selected and the test criterion *α* = 0.05. *P* < 0.05 was considered statistically significant between the groups.

## 3. Results

### 3.1. Comparison of General Information among the Three Groups

The differences were not statistically significant (*P* > 0.05) when comparing the gender, age, time of surgery, body mass index, etiology, PLT, Hb, PT, TT, FIB, and APTT in the three groups (Table 1).

### 3.2. Comparison of Postoperative Recovery-Related Indexes among the Three Groups

The differences were statistically significant (*P* < 0.05) when comparing the postoperative time to the bed activity, the hospital stay, and the incidence of postoperative adverse reactions in the three groups. Among them, the postoperative bed activity time, the hospitalization time, and the incidence of postoperative adverse reactions in the combined group and FTS group were lower than those in the regular group, and the postoperative bed activity time in the combined group was lower than that in the FTS group (*P* < 0.05, Figure 1).

The article "Analysis of Fast-Track Surgery with Pain Care on Postoperative Pain Improvement and Complication Prevention in Perioperative Spine Surgery Patients" was published in 2022. Journal: Emerg Med Int.

### 3.3. Comparison of Pain Scores at Different times among the Three Groups

The differences were statistically significant (*P* < 0.05) when comparing the NRS scores at different times after surgery in the three groups. Among them, the NRS scores at 12 h, 24 h, 48 h, and 72 h postoperatively in the combined group and FTS group were lower than those in the regular group, and the NRS scores at 12 h and 24 h postoperatively in the combined group were lower than those in the FTS group (*P* < 0.05, Figure 2).

### 3.4. Comparison of Pain Levels among the Three Groups at Different times

The differences were statistically significant (*P* < 0.05) when comparing the pain levels of the three groups at 12 h, 24 h, and 48 h postoperatively. Among them, the pain level at 12 h postoperatively in the combined group was lower than that in the conventional group, and the pain levels at 24 h and 48 h postoperatively in both the FTS group and the combined group were lower than those in the conventional group; the pain level at 24 h postoperatively in the combined group was lower than that in the FTS group (*P* < 0.05). The differences in the NRS scores at 72 h postoperatively were not statistically significant in any of the three groups (*P* > 0.05, Table 1).

### 3.5. Comparison of Complications among the Three Groups

The total complication rates of postoperative bleeding, postoperative pressure sores, urinary retention, and incisional infections were statistically significant (*P* < 0.05) when compared among the three groups. The total complication rates in the FTS and combined groups were lower than those in the conventional group (*P* < 0.05), and the differences between the FTS and combined groups were not significant (*P* > 0.05, Table 2).

### 3.6. Comparison of Nursing Satisfaction among the Three Groups

When comparing the nursing satisfaction of the three groups, the differences were statistically significant (*P* < 0.001), in which the nursing satisfaction of the FTS group and the combined group were higher than that of the conventional group, and the nursing satisfaction of the combined group was higher than that of the FTS group (*P* < 0.05, Table 3).

## 4. Discussion

Patients after spinal surgery need absolute bed rest after surgery due to the special location of the lesion, which restricts patients' activities to a certain extent. At the same time, the body will be in a state of stress when the patient is subjected to various physical or chemical injuries or is in a large emotional fluctuation, in which the patient's neurological and endocrine functions and the internal environment of the body will undergo certain changes, resulting in pain, fatigue, nausea and vomiting, immune dysfunction, and other external manifestations [13, 14]. Among them, pain is the most common irritant in orthopedic clinics. Pain is a negative emotional experience caused by tissue damage or potential tissue damage and is an important vital sign in addition to pulse, blood pressure, temperature, and respiration during surgical treatment [15]. Postoperative pain can easily lead to patients' irritability, anxiety, and other negative emotions and has a serious impact on the quality of sleep and postoperative rehabilitation of patients, which in turn leads to delayed discharge events of patients undergoing surgery, as well as unscheduled visit and admission events after discharge. Therefore, nursing staff should carry out various interventions for patients after surgery [16, 17].

The article "Analysis of Fast-Track Surgery with Pain Care on Postoperative Pain Improvement and Complication Prevention in Perioperative Spine Surgery Patients" was published in 2022. Journal: Emerg Med Int.

The results showed that the NRS scores of the combined group and FTS group at each time point after surgery were lower than those of the conventional group, and the NRS scores of the combined group at 12 h and 24 h after surgery were lower than those of the FTS group (*P* < 0.05). FTS is a collaborative therapeutic intervention system, and FTS-based care management aims to reduce surgical stress and postoperative complications and accelerate postoperative recovery of patients; this care model is highly adaptable in the application of various surgical care processes [18]. In addition to helping patients get a comfortable position, removing various factors that induce pain aggravation, and creating a good hospital environment through routine nursing, special pain care also provides preoperative and postoperative pain education through brochures, videos, etc. Patients' mastery of the concept of postoperative pain can help patients understand the pain evaluation methods, report pain timely and accurately, master self pain relief methods, and strengthen pain control [19, 20]. Through psychological care to ease patients' fear and anxiety and other psychological aspects, we give patients appropriate emotional support such as sympathy and comfort so that patients can maintain a relaxed and stable mood and improve their pain threshold. Through multimodal, individualized, and timely administration of analgesic programs, an individualized and reasonable analgesia is administered according to the patient's pain level, effectively relieving patients' pain discomfort [21, 22].

In this study, the ambulation time, hospital stay, and incidence of adverse reactions and complications after surgery in the combined group and FTS group were shorter or lower than those in the conventional group, and the ambulation time after surgery in the combined group was shorter than that in the FTS group (*P* < 0.05). These results indicated that combined nursing was better than FTS management in reducing perioperative pain severity, shortening postoperative rehabilitation time, and reducing the incidence of adverse reactions and complications in spine surgery. In this study, our nursing staff formed an FTS nursing team to optimize the traditional perioperative care methods in spine surgery, develop a professional nursing plan, and combine FTS theory in the nursing process to provide special care for patients, including preoperative education, targeted intraoperative care, and rapid postoperative rehabilitation, to relieve patients' preoperative tension through comprehensive management, encourage patients to get out of bed early on the basis of adequate postoperative pain relief, improve patients' ability to take care of themselves, and promote rapid recovery.

The article "Analysis of Fast-Track Surgery with Pain Care on Postoperative Pain Improvement and Complication Prevention in Perioperative Spine Surgery Patients" was published in 2022. Journal: Emerg Med Int.

In addition, the nursing satisfaction levels in the combined group and FTS group were higher than that in the routine group, and the nursing satisfaction level in the combined group was higher than that in the FTS management group (*P* < 0.05). The possible reason why combined care can improve patients' satisfaction with nursing care may be the addition of pain-specific care on top of FTS, and comprehensive care is carried out for patients under the guidance of personalized and holistic thinking. This not only relieves patients' bad emotions but also improves patients' pain, postoperative adverse reactions, and complications and accelerates the rehabilitation process, thus improving their satisfaction with nursing work [23, 24].

In conclusion, FTS care combined with pain-specific care for spine surgery patients can effectively relieve patients' pain discomfort, shorten their hospital stay, and improve patient satisfaction.

## Figures and Tables

**Figure 1:** Comparison of postoperative recovery-related indexes among the three groups. *Note*. Comparison with the regular group, ^*∗*^*P* < 0.05. Comparison with the FTS group, ^#^*P* < 0.05.

**Figure 2:** Comparison of pain scores at different times among the three groups. *Note*. Comparison with the regular group, ^*∗*^*P* < 0.05. Comparison with the FTS group, ^#^*P* < 0.05.

**Table 1:** Comparison of pain levels among the three groups at different times (*n*, %).

Group/time	Regular group (*n* = 42)			FTS group (*n* = 42)			Combined group (*n* = 42)		
	Mild	Moderate	Severe	Mild	Moderate	Severe	Mild	Moderate	Severe
Pre-op	0 (0.00)	16 (38.10)	26 (61.90)	0 (0.00)	19 (45.24)	23 (54.76)	0 (0.00)	16 (38.10)	26 (61.90)
12 h post-op	1 (2.38)	37 (88.10)	4 (9.52)	2 (4.76)	39 (92.86)	1 (2.38)	7 (16.67)^*∗*^	35 (83.33)	0 (0.00)
24 h post-op	11 (26.19)	31 (73.81)	0 (0.00)	22 (52.38)^*∗*^	20 (47.62)	0 (0.00)	35 (83.33)^*∗*#^	7 (16.67)	0 (0.00)
48 h post-op	21 (50.00)	21 (50.00)	0 (0.00)	37 (88.10)^*∗*^	5 (11.90)	0 (0.00)	38 (90.48)^*∗*^	4 (9.52)	0 (0.00)
72 h post-op	38 (90.48)	4 (9.52)	0 (0.00)	42 (100.00)	0 (0.00)	0 (0.00)	42 (100.00)	0 (0.00)	0 (0.00)

*Note.* Comparison with the regular group, ^*∗*^*P* < 0.05. Comparison with the FTS group, ^#^*P* < 0.05.

The article "Analysis of Fast-Track Surgery with Pain Care on Postoperative Pain Improvement and Complication Prevention in Perioperative Spine Surgery Patients" was published in 2022. Journal: Emerg Med Int.

**Table 2:** Comparison of complications among the three groups (*n*, %).

Group	Postoperative bleeding	Postoperative pressure sores	Urinary retention	Incisional infections	Total
Regular group (*n* = 42)	1 (2.38)	2 (4.76)	4 (9.52)	4 (9.52)	11 (26.19)
FTS group (*n* = 42)	1 (2.38)	0 (0.00)	1 (2.38)	2 (4.76)	4 (9.52)^*∗*^
Combined group (*n* = 42)	0 (0.00)	1 (2.38)	1 (2.38)	1 (2.38)	3 (7.14)^*∗*^
*χ* ^*2*^ value					7.389
*P* value					0.025

**Table 3:** Comparison of nursing satisfaction among the three groups (*n*, %).

Group	Satisfied	Quite satisfied	Dissatisfied	Total
Regular group (*n* = 42)	9 (21.43)	22 (52.38)	11 (26.19)	31 (73.81)
FTS group (*n* = 42)	21 (50.00)	17 (40.48)	4 (9.52)	38 (90.48)^*∗*^
Combined group (*n* = 42)	28 (66.67)	14 (33.33)	0 (0.00)	42 (100.00)^*∗*#^
*χ* ^*2*^ value				14.076
*P* value				<0.001

## Data Availability

The data are available from the corresponding author upon request.
